The article "Tripartite motif-containing 14 (TRIM14) promotes epithelial-mesenchymal transition via ZEB2 in glioblastoma cells" was retracted in 2023. Reasons: manipulated images; signs of a paper mill; unreliable results or conclusions; lack of ethics approval or compliance.

# Tripartite motif-containing 14 (TRIM14) promotes epithelial-mesenchymal transition via ZEB2 in glioblastoma cells

**DOI:** 10.1186/s13046-019-1070-x

**Published:** 2019-02-06

**Authors:** Shuang Feng, Xiaomin Cai, Yangyang Li, Xiaoguang Jian, Linxin Zhang, Bin Li

**Affiliations:** 1 Department of Encephalopathy, The Third Affiliated Hospital of Nanjing University of Chinese Medicine, Nanjing, Jiangsu China; 2 Department of Neurosurgery, The First Affiliated Hospital of Nanjing Medical University, Nanjing, Jiangsu China

**Keywords:** Glioblastoma, TRIM14, ZEB2, Invasion, Ubiquitination

## Abstract

**Background:**

Several members of the tripartite motif-containing (TRIM) protein family have been reported to serve as vital regulators of tumorigenesis. Recent studies have demonstrated an oncogenic role of TRIM 14 in multiple human cancers; however, the importance of this protein in glioblastoma remains to be elucidated.

**Methods:**

The expression levels of TRIM14 were analyzed in a series of database and were examined in a variety of glioblastoma cell lines. Two independent TRIM14 shRNA were transfected into LN229 and U251 cells, and the effect of TRIM14 depletion was confirmed. Transwell assay and wound healing assay assay were carried out to assess the effect of TRIM14 depletion on glioblastoma cell invasion and migration. Western blotting was performed to screen the downstream gene of TRIM14. The stability analysis and Ubiquitylation assays and Orthotopic xenograft studies were also performed to investigate the role of TRIM14 and the relationship with downstream gene. Human glioblastoma tissues were obtained and immunohistochemical staining were carried out to confirm the clinical significance of TRIM14.

**Results:**

In this study, we showed that TRIM14 was upregulated in human glioblastoma specimens and cell lines, and correlated with glioblastoma progression and shorter patient survival times. Functional experiments showed that decreased TRIM14 expression reduced glioblastoma cell invasion and migration. Furthermore, we identified that zinc finger E-box binding homeobox 2 (ZEB2), a transcription factor involved in epithelial–mesenchymal transition, is a downstream target of TRIM14. Further investigation revealed that TRIM14 inactivation significantly facilitated ZEB2 ubiquitination and proteasomal degradation, which led to aggressive invasion and migration. Our findings provide insight into the specific biological role of TRIM14 in tumor invasion.

**Conclusions:**

Our findings provide insight into the specific biological role of TRIM14 in tumor invasion, and suggest that targeting the TRIM14/ZEB2 axis might be a novel therapeutic approach for blocking glioblastoma.

**Electronic supplementary material:**

The online version of this article (10.1186/s13046-019-1070-x) contains supplementary material, which is available to authorized users.

## Background

Glioblastoma is the most common and aggressive tumor of the nervous system. Despite intensive treatment with combined multiagent chemotherapy and surgery, patients generally show poor prognosis and incurable relapse of the disease [1–3]. The median survival time of patients with glioblastoma is short, at approximately 14.6 months [4, 5]. Therefore, effective identification and development of novel molecular approaches to the diagnosis, treatment and prognosis of patients with glioblastoma remain urgent clinical requirements.

The tripartite motif-containing (TRIM) family proteins are defined by a conserved domain architecture composed of three zinc-binding regions: a RING finger, one or two B-boxes, and a coiled-coil domain. Accumulating evidence indicates that TRIM family proteins play important roles in various physiological processes, including cell proliferation, migration, invasion, apoptosis and differentiation, and the cell cycle [6–8]. TRIM14, which is located at chromosome 9q22, is a member of the TRIM family and was first discovered as being overexpressed in HIV-infected human and simian lymphomas by subtractive hybridization [9–11]. Subsequent studies revealed that TRIM14 may undergo amplification in tongue squamous cell carcinoma and non-small cell lung cancer cells [12, 13]. Later, researches of TRIM14 in a wide variety of tumor were also reported. TRIM14 promotes the migration and invasion of gastric cancer [14].

TRIM14 promotes breast cancer cell proliferation by inhibiting apoptosis [15]. TRIM14 regulates cell proliferation and invasion in osteosarcoma via promotion of the AKT signaling pathway [16].However, the expression levels and biological functions of TRIM14 in glioblastoma remain to be elucidated.

Epithelial–mesenchymal transition (EMT) is a key process that occurs during the development of organisms and the progression of epithelial tumors to metastatic cancers [17, 18]. EMT involves disruption of the cytoskeleton, intercellular adhesions and normal expression of transcriptional factors, and may be an important factor contributing to glioblastoma tumorigenesis, metastasis, and chemotherapy resistance [19–23]. EMT is driven by a network of embryonic EMT-inducing transcription factors (EMT-TFs), which include members of several protein families such as ZEB1, Snial1, Slug, and Twist1, [24–28]. Growing evidence has revealed that EMT-TFs play critical roles, directly or indirectly, in embryogenesis and cancer initiation and progression [29–31]. Moreover, EMT is regulated by several key transcription factors, which in the structures of zinc finger protein and basic helix-loop-helix (bHLH), including ZEB family members [25]. However, the complex molecular network and various mechanistic steps involved in these effects remain ambiguous. Here, we identified upregulation of TRIM14 in glioblastoma tissues and cell lines, and found that ectopic TRIM14 expression induced glioblastoma cell invasion and migration. Furthermore, we found that deletion of TRIM14 suppressed zinc finger E-box binding homeobox 2 (ZEB2) levels post-translationally through effects on the ubiquitin–proteasome pathway. ZEB2 (also known as SIP1) is a member of the ZEB family of 2-handed zinc finger/homeodomain proteins [32]. Recent reports highlighted that ZEB2 is closely related to EMT, thus suggesting that ZEB2 is a key factor in promoting tumor initiation and development [33–35]. Our data demonstrate that TRIM14 functions as a novel regulator of EMT by controlling the abundance of the key transcription factor ZEB2.

## Methods

### Human tissue samples

Fifty two GBM tissue specimens were obtained by the Department of Neurosurgery, the First Affiliated Hospital of Nanjing Medical University. Ten normal brain tissues were collected as a negative control from patients undergoing decompressive craniotomy for traumatic brain injury in the First Affiliated Hospital of Nanjing Medical University. The histological features of all the specimens were identified by pathologists according to the WHO criteria. All patients gave written informed consent for the studies before surgery excision. This study was approved by the institutional review board and the ethics committee of Nanjing Medical University, and written informed consent was obtained from all patients.

### Cell culture and reagents

The human GBM cell lines LN229, A172, LN229, U118 were purchased from the American Type Culture Collection (ATCC). The human GBM cell lines U251 and T98G were obtained from RIKEN bioresource center (Tsukuba, Japan). To maintain authenticity of the cell lines, frozen stocks were prepared from initial stocks, and every 3 months, a new frozen stock was used for the experiments. For each experiment, GBM cells were sustained in Dulbecco’s modified Eagle’s medium (DMEM) supplemented with 10% fetal bovine serum and 1% penicillin/streptomycin. Sodium pyruvate, nonessential amino acids, L-glutamine, and a vitamin solution. NHAs were purchased from Lonza (Walkersville, MD) and maintained following the manufacturer’s instructions.

ShTRIM14, shCtrl, shZEB2, pLVGFP- TRIM14 and pLVGFP- TRIM14 vector were purchased from GenePharma (Shanghai, China). All the plasmids were transfected into cells grown in DMEM culture media using Lipofectamine 3000 Transfection Reagent (Invitrogen, Carlsbad, CA) according to the manufacturer’s instructions.

### RNA extraction and qRT-PCR analysis

The total RNA from cell or tissues lines was was extracted using TRIzol Reagent (Invitrogen) following the manufacturer’s protocol. qRT- PCR was performed using an Applied Biosystems 7900 Sequence Detection system. First-strand cDNA was synthesized using the Primerscript RT Master Mix (TaKaRa). Primers used in qRT-PCR experiments were as follows: Tripartite motif-containing 14 (TRIM14): 5′-GCAGAAACTCAGCCAAGAA-3′ and 5′-CTTGACTCTGCATTAGCCT-3′, Zinc finger E-box binding homeobox 2 (ZEB2): 5′-GGCGCAAACAAGCCAATCCCA-3′ and 5′-TTCACTGGACCATCTACAGAGGCTT-3′, Glyceraldehyde 3-phosphate dehydrogenase (GAPDH) mRNA was also amplified in the same PCR reactions as an internal control using the primers 5’-TGCACCACCAACTGCTTAGC-3′ and 5’-GGCATGGACTGTGGTCATGAG-3′. Relative gene expression was calculated via 2^-ΔΔC^_t_ method.

### Western blotting assay

Western blotting assay was performed as previously described. Briefly, cells were lysed in RIPA buffer.Protein concentrations were detected with the BCA protein assay (Pierce, Waltham, MA, USA), and equal amounts of protein (20μg) were separated by 10% SDS-PAGE followed by electro-transfer onto a polyvinylidene difluoridemembrane (PVDF, Millipore, MA, USA). The membranes were blocked for 2h with 5% nonfat milk and then incubated at room temperature with primary antibodies. After extensive wash in TBS-Tween (3 × 5 min), the membrane was incubated with a horseradish peroxidase-conjugated secondary antibody directed to the correct primary antibody species. The bound antibody complexes were detected by using the enhanced chemiluminescence method (Amersham Biosciences, Uppsala, Sweden). After detection, the membrane is stripped in stripping buffer, and re-blotted for β-actin. The signal of β-actin was used as an internal control to normalize the band intensity. Digitized band signal was generated by a scanner (Microtek 9800XL), and analyzed using NIH Image J. The following antibodies used in this study were purchased from Abcam: TRIM14 (ab185349), N-cadherin (ab18203), E-cadherin (ab1416), Vimentin (ab8978), Snail1 (ab53519), Twist1 (ab50581), ZEB1 (ab203829), SLUG (ab27568), Anti-Myc(ab32), Anti-Flag (ab1238) and β-actin (ab8227). ZEB2 (NBP1–82991) was purchased from Novus. HA (#3724) was purchased from CST.

### Invasion assay

Invasion capacity was assessed using 24-well BD Matrigel invasion chambers (BD Biosciences) according to the manufacturer’s instructions. 2 × 10^4^ cells were seeded in the upper well of the invasion chamber in DMEM without serum. The lower chamber well contained DMEM supplemented with 10% FBS to stimulate invasion. After incubation for 24 h, non-invading cells were removed from the top well with a cotton swab while the bottom cells were fixed with 100% methanol, and stained with 0.1% crystal violet, and photographed in three independent 10× magnification fields.capacity.

### Wound healing assay

About 3 × 10^5^ cells were seeded in 6-well dishes and an incision was made in the central area of the confluent culture to create an artificial wound. Images of the wound area were captured by microscope (Leica, Wetzlar, Germany) 24 h after injury. Cells grown into the scratched center area were manually counted.

### 3D spheroid BME cell invasion assays

Established cell lines and the transfected were cultured to 70% confluence. Cells were seeded at a 0.2 × 10^5^ cells/ml density in 96-well ultralow adherence plates (#7007, Costar). Over the course of 96 h these cells were induced to aggregate into a multicellular spheroid with an estimated density of 2000 cells and then matrigel was added into wells. After 48 h, motion of cells was confirmed as fully formed under light microscopy.

### IHC assay

The IHC assay was conducted on human GBM tissue. Fresh human GBM tissue were under cryopreservation and processed into frozen sections. Five-micronthick sections were immunohistochemical staining with streptavidin-biotin immunoperoxidase assay was performed using special antibodies against TRIM14 and ZEB2. Slides were imaged under a light microscope (Leica, German) at 200 or 400 × magnification.

### Orthotopic xenograft studies

Orthotopic xenograft experiments were approved by the Animal Management Rule of the Chinese Ministry of Health(documentation 55, 2001). LN229 cells (2 × 10^6^) transfected with shCtrl and shTRIM14 were subcutaneously injected into 36-day-old male nude mice (Cancer Institute of the Chinese Academy of Medical Science). 10 days after injection, the tumor was visible. And within 8 weeks, all the male nude mice were sacrificed and the tumor tissues were excised and frozen immediately at − 80°C for further study.

### Statistical analysis

Data were analyzed via one-way analysis of variance (ANOVA) for multiple group comparisons and two tailed student’s *t*-tests for two-group comparisons after passed normality test. Mann-Whitney non-parametric test was used when data did not follow normal distribution. Statistics was conducted using SPSS 13.0 soft package. Differences were considered statistically significant at *p* < 0.05.

## Results

### TRIM14 levels are increased in glioblastoma tissues

To investigate the potential function of TRIM14 in glioblastoma, we analyzed TRIM14 in samples from a cohort of 62 patients, including 10 normal brain tissue samples and 52 glioblastoma samples of different grades, by quantitative reverse transcription PCR (qRT-PCR). As shown in Fig. 1a, there was a marked positive correlation between TRIM14 expression and patient clinical grade. Next, we assessed TRIM14 protein levels in glioblastomas of different grades by western blotting (Fig. 1b). The results were consistent with those of qRT-PCR. We also compared the TRIM14 protein levels in these primary glioblastoma tissues with those in paired normal brain tissues by western blotting, and found that TRIM14 expression was considerably upregulated in glioblastomas compared with normal brain tissue (Fig. 1c). Next, we analyzed TRIM14 levels in normal human astrocytes (control) and six glioma cell lines (U87, U251, U118, LN229, T98G and HS683) using qRT-PCR. All six glioblastoma cell lines exhibited significantly higher TRIM14 mRNA expression than the normal human astrocytes, and TRIM14 was particularly highly expressed in LN229 and U251 cells (Fig. 1d). Immunohistochemistry assays indicated that TRIM14 expression was lowest in normal tissues and gradually upregulated as glioma malignancy grade increased(Fig. 1e). To further determine whether the high TRIM14 expression level was a universal phenomenon in glioblastoma patients, we analyzed TRIM14 expression in glioblastoma specimens and normal brain tissues using three datasets: TCGA, REMBRANDT, and GEO (GSE16011). As shown in Additional file 1: Figure S1A, TRIM14 expression levels were consistently increased in glioblastoma specimens compared with normal brain tissues in all three of these individual databases (REMBRANDT *P* < 0.0001; GSE16011 *P* = 0.0106; TCGA *P* < 0.0001). The dramatic upregulation of TRIM14 in glioblastoma tissues led us to consider whether TRIM14 expression might correlate closely with glioblastoma patient prognosis. We therefore conducted Kaplan–Meier survival analysis using the data from the three databases. We found that patients with low TRIM14 levels exhibited much longer overall survival than those with high TRIM14 expression levels (Additional file 1: Figure S1B, REMBRANDT *P* = 0.0469; GSE16011 *P* = 0.0340; TCGA *P* = 0.0489). This suggests that TRIM14 could be used as a prognostic biomarker in patients with glioblastoma. Taken together, these results suggest that TRIM14 is increased in both glioblastoma tissues from patients and in cell lines, compared with normal brain tissues and cells, and may play a vital role in tumorigenesis and malignancy.

**Fig. 1:** TRIM14 is increased in GBM tissues and cell lines. **a** Comparison of TRIM14 levels between normal brain tissues (NBT) and different grade glioblastoma specimens using qRT-PCR analysis. *p < 0.05; **p < 0.01; ***p < 0.001. **b** Western blot analysis of TRIM14 protein expression in different grade glioblastoma tissue and normal brain tissue. **c** Western blotting analysis of TRIM14 protein in 6 GBM samples and matched normal tissues. (*N* = normal tissues,T = GBM) (**d**) qPCR analysis of TRIM14 expression in 6 glioma cell lines as well as NHA controls. 6 cell lines show significantly increased TRIM14 protein levels. *p < 0.05; ***p < 0.001, *n* = 3 experiments. **e** The expression of TRIM14 is tested in normal brain tissues and glioma tissues (I-IV grade) from Jiangsu Province Hospital by Immunohistochemistry

### Reduced TRIM14 expression suppresses tumor invasion and migration

To further investigate the effect of TRIM14 on the tumorigenesis and malignancy of human glioblastoma cells, we performed in vitro loss-of-function analysis by knocking down TRIM14 with two short hairpin RNA (shRNA) targeting TRIM14 (shTRIM14) in two glioblastoma cell lines. To confirm the knockdown efficiency, western blot analysis was performed; this verified that TRIM14 protein levels were remarkably decreased in both LN229 and U251 cells transfected with shTRIM14 compared with those transfected with a scrambled control shRNA. Furthermore, we found that in both LN229 and U251 cells, TRIM14 knockdown significantly increased levels of the epithelial biomarker E-cadherin, and simultaneously decreased levels of the mesenchymal biomarkers N-cadherin and Vimentin (Fig. 2a). A transwell invasion cassay was conducted to investigate the influence of TRIM14 on invasion and migration ability in glioblastoma. Silencing TRIM14 expression by shRNA significantly reduced LN229 and U251 cell invasiveness (***p < 0.001, *n* = 3, Fig. 2b). Next, a wound healing assay was performed using shTRIM14-transfected LN229 and U251 cells, and corresponding control cells. Knockdown of TRIM14 markedly suppressed the migration of LN229 and U251 cells into the scratch-wounded area (***p < 0.001, *n* = 3, Fig. 2c), and the statistical data was in Fig. 2d. Moreover, this conclusion was confirmed by 3D spheroid BME cell invasion assays (***p < 0.001, *n* = 3, Fig. 2e and f). Further, we evaluate the effect of TRIM14 inhibition on proliferation by CCK-8 assays and colony formation assays. As shown in Additional file 2: Figure S2A and B(***p < 0.001, *n* = 3), although downregulating TRIM14 by two shTRIM14 showed no statistical influence on cell proliferation in the first three days, but significantly reduced cell proliferation of LN229 and U251 cell after 5 days, indicating that TRIM14 also had potential abilities to promote the glioma cell growth(***p < 0.001, *n* = 3, Additional file 2: Figure S2B). Collectively, these results indicate that TRIM14 enhances invasion and migration of glioblastoma cancer cells by promoting EMT.

**Fig. 2:** TRIM14 increases migration/invasion in GBM cells by EMT. **a** Western blot analysis of TRIM14, N-cadherin, E-cadherin and Vimentin in LN229 and U251 cells transduced with shTRIM14–1, shTRIM14–2 or control shRNA. Equal loading is confirmed by β-actin levels. **b** Representative images of transwell invasion assay using LN229 and U251 cells transfected with the indicated shRNA. Quantification of transwell invasion assay is shown. ***p < 0.001; *n* = 3 experiment. **c**-**d** Representative images of wound healing assay using LN229 and U251 cells with the indicated shRNA. Quantification of wound healing assay is shown. ***p < 0.001, *n* = 3 experiments. **e**-**f** Representative images of 3D spheroid BME cell invasion assays using LN229 and U251 cells with the indicated shRNA. Quantification of 3D spheroid BME cell invasion assays is shown. ***p < 0.001, *n* = 3 experiments

### Exogenous TRIM14 expression promotes tumor invasion and migration

Next, two glioma cell lines, HS683 and U87, were selected to investigate malignant phenotypic changes following TRIM14 overexpression. HS683 and U87 glioma cell lines were transduced with a lentivirus carrying TRIM14 to form stable TRIM14-overexpressing cell lines. Western blot analysis showed that TRIM14-overexpressing significantly increased levels of the mesenchymal biomarkers N-cadherin and Vimentin, and levels of the epithelial biomarker E-cadherin were remarkably decreased(Fig. 3a). We performed transwell invasion assay and wound healing assay after transfecting cells. We detected significant promoting effects on the invasion and migration of HS683 and U87 cells lines(***p < 0.001, *n* = 3, Fig. 3b and c). The statistical results were shown in Fig. 3b and d. Further, when we used 3D spheroid BME cell invasion assays to evaluate the effect of TRIM14 on invasion, the results were similar to those acquired using the transwell invasion assays and wound healing assays(***p < 0.001, *n* = 3, Fig. 3e and f). CCK-8 assays and Colony formation assays were performed after transfecting with the lentivirus(***p < 0.001, *n* = 3, Additional file 2: Figure S2C and D). We detected significant promoting effects on the viabilities of HS683 and U87 cells compared with the controls. Taken together, these data demonstrated that TRIM14 mediates glioma cell EMT processes and proliferation.

**Fig. 3:** TRIM14 overexpression promotes migration/invasion in glioma cells by EMT. **a** Western blot analysis of TRIM14, N-cadherin, E-cadherin and Vimentin in HS683 and U87 cells transduced with vector or TRIM14. Equal loading is confirmed by β-actin levels. **b** Representative images of transwell invasion assay using HS683 and U87 cells transfected with vector or TRIM14. Quantification of transwell invasion assay is shown. ***p < 0.001; *n* = 3 experiment. **c**-**d** Representative images of wound healing assay using HS683 and U87 cells with vector or TRIM14. Quantification of wound healing assay is shown. ***p < 0.001, *n* = 3 experiments. **e**-**f** Representative images of 3D spheroid BME cell invasion assays using HS683 and U87 cells with vector or TRIM14. Quantification of 3D spheroid BME cell invasion assays is shown. ***p < 0.001, *n* = 3 experiments

### ZEB2 inhibition is involved in the TRIM14 knockdown-induced reduction in invasion and migration ability

To explore the TRIM14-independent mechanisms underlying the increased invasiveness and migration, we used LN229 and U251 cells to evaluate whether TRIM14 knockdown affected the EMT-inducing transcription factors Snail1, Twist1, ZEB1, ZEB2 and SLUG, which are known to play a role in EMT and tumorigenesis After TRIM14 was knocked down in both LN229 and U251 cell lines with two shRNAs, only ZEB2 levels were markedly decreased (Fig. 4a). This led us to hypothesize that the effects of TRIM14 on EMT were dependent on ZEB2. In cells in which TRIM14 expression was silenced, the alterations in EMT biomarkers were reversed by ZEB2 overexpression (Fig. 4b). We also conducted wound healing assays and transwell invasion assays to demonstrate the function of ZEB2 in TRIM14-independent invasion and migration. Importantly, we found that upregulation of ZEB2 completely restored the invasive capacity of LN229 and U251 cells inhibited by shTRIM14 (***p < 0.001, *n* = 3, Fig. 4c and d). This was consistent with the results of 3D spheroid BME cell invasion assays ((***p < 0.001, *n* = 3, Fig. 4e). For further exploration the relationship of ZEB2 and TRIM14, we detected the changes after overexpressing TRIM14 in HS683 and U87 cells line. Western blot analysis showed that ZEB2 was increased after TRIM14 overexpressing (Fig. 5a), but other EMT-inducing transcription factors showed no change. And the EMT biomarkers altered by exogenous TRIM14 expression were reversed after ZEB2 inhibition by shZEB2 (Fig. 5b). In line with those properties, TRIM14 significantly promoted cell invasion and migration in HS683 and U87 while ZEB2 inhibition significantly reversed this experimental phenomena by using wound healing assays and transwell invasion assays (***p < 0.001, *n* = 3, Fig. 5c and d). In addition, 3D spheroid BME cell invasion assays also showed the increased ability of invasion and migration by ectopical expression of TRIM14 were reversed after transfected with shZEB2 (***p < 0.001, *n* = 3, Fig. 5e). These findings further support the possibility that ZEB2 might be a downstream and direct functional target of TRIM14.

**Fig. 4:** ZEB2 is a downstream target of TRIM14. **a** Western blot analysis of TRIM14, EMT related biomarks (Snail1, Twist1, ZEB1, ZEB2 and SLUG), and β-actin in LN229 and U251 cells transfected with shTRIM14–1, shTRIM14–2 or control shRNA. **b** Western blot analysis of TRIM14, N-cadherin, E-cadherin, Vimentin and β-actin in LN229 and U251 cells transduced with the indicated plasmid. **c** Representative images of transwell invasion assay using LN229 and U251 cells transfected with the indicated plasmid. Quantification of transwell invasion assay is shown. ***p < 0.001; *n* = 3 experiment. **d** Representative images of wound healing assay using LN229 and U251 cells with the indicated plasmid. Quantification of wound healing assay is shown. ***p < 0.001, *n* = 3 experiments. **e** Representative images of 3D spheroid BME cell invasion assays using LN229 and U251 cells with the indicated plasmid. Quantification of 3D spheroid BME cell invasion assays is shown. ***p < 0.001, *n* = 3 experiments

**Fig. 5:** ZEB2 is involved in the function of TRIM14. **a** Western blot analysis of TRIM14, EMT related biomarks (Snail1, Twist1, ZEB1, ZEB2 and SLUG), and β-actin in HS683 and U87 cells transfected with vector or TRIM14. **b** Western blot analysis of TRIM14, N-cadherin, E-cadherin, Vimentin and β-actin in HS683 and U87 cells transduced with the indicated plasmid. **c** Representative images of transwell invasion assay using HS683 and U87 cells transfected with the indicated plasmid. Quantification of transwell invasion assay is shown. ***p < 0.001; *n* = 3 experiment. **d** Representative images of wound healing assay using HS683 and U87 cells with the indicated plasmid. Quantification of wound healing assay is shown. ***p < 0.001, *n* = 3 experiments. **e** Representative images of 3D spheroid BME cell invasion assays using HS683 and U87 cells with the indicated plasmid. Quantification of 3D spheroid BME cell invasion assays is shown. ***p < 0.001, *n* = 3 experiments

### Reduced TRIM14 expression correlates with ZEB2 polyubiquitination and proteasomal degradation

Next, we explored how TRIM14 affects ZEB2 expression. We identified no obvious differences in ZEB2 mRNA expression between control cells and cells with TRIM14 knocked down (***p < 0.001, *n* = 3, Fig. 6a). This ruled out the possibility that TRIM14 regulates ZEB2 expression at the mRNA level, and suggested that it might affect ZEB2 protein stability. Addition of the proteasome inhibitor MG132 reversed the decrease in ZEB2 levels after TRIM14 depletion (Fig. 6b). We next examined the effect of TRIM14 depletion on the stability of endogenous ZEB2 protein in the presence of cycloheximide, an inhibitor of protein translation. Short- and long-duration exposures of ZEB2 protein by western blotting showed that ZEB2 was degraded more rapidly in TRIM14-knockdown cells compared with control cells (***p < 0.001, *n* = 3, Fig. 6c). Quantification of the bands on the western blots revealed a rapid decline in ZEB2 levels after TRIM14 depletion by small interfering RNA targeting TRIM14.

**Fig. 6:** Depletion of TRIM14 increased ZEB2 polyubiquitination and proteasomal degradation. **a** qTR-PCR analysis of TRIM14 and ZEB2 mRNA level in LN229 and U251 cells after TRIM14 knowdown by shTRIM14. Depletion of TRIM14 does not alter ZEB2 mRNA. ***p < 0.001, *n* = 3 experiments. **b** Western blot analysis of TRIM14, ZEB2 and β-actin in LN229 and U251 cells transduced with the indicated shRNA in the absence or presence of 10μM MG132. **c** LN229 and U251 cells transfected with shTRIM14 were treated with cycloheximide (100μg/ml, pretreated for 15 min and for varying durations), and collected at the indicated times for western blot. Quantification of ZEB2 expression relative to β-actin is shown. Results are shown as mean ± standard deviation. *n* = 3 independent experiments. ***, *P* < 0.001, two-way ANOVA test. **d** LN229 and U251 cells transfected with HA-UB and the indicated shRNA were treated with MG132 for 8 h before harvest. ZEB2 was immunoprecipitated with anti-ZEB2 antibody and immunoblotted with anti-HA antibody. **e** LN229 and U251 cells were transduced with the indicated shRNA for 48 h, treated with the proteasome inhibitor MG132 for 6 h, and then subjected to analysis of ZEB2 ubiquitination and IB analyses. **f** HS683 and U87 cells were transduced with the Myc-TRIM14, Flag-FBXO45 or vector control for 48 h, treated with the proteasome inhibitor MG132 for 6 h, and then subjected to analysis of ZEB2 ubiquitination and IB analyses

Ubiquitin is a crucial post-translational modification involved in proteasomal degradation. The stability of ZEB family members is known to be regulated by the ubiquitin–proteasome system. Therefore, we investigated whether TRIM14 altered the stability of ZEB2 by affecting the ubiquitin–proteasome system. Ubiquitylation assays were carried out to determine whether TRIM14 mediates ZEB2 proteolysis via the ubiquitin pathway (Fig. 6d). We found that reducing TRIM14 expression significantly increased ZEB2 polyubiquitylation. Our results suggest that TRIM14 determines the stability of ZEB2 by mediating its proteasomal degradation via polyubiquitination. F-Box protein 45(FBXO45) function as an ubiquitin E3 ligase to regulate ZEB2 protein stability at the posttranslational level. FBXO45 play a vital role in facilitating ZEB2 ubiquitination in glioma cells. This suggests that TRIM14 have an antagonistic role to oppose FBXO45-mediated ubiquitination of ZEB2. To further validate this hypothesis, we reconstituted a regulatory system by overexpressing TRIM14 with FBXO45 or knocking down TRIM14 and FBXO45 to directly assess ZEB2 expression. As shown in Fig. 6e, TRIM14 downregulation increased ZEB2 ubiquitination, whereas FBXO45 knockdown reduced ZEB2 ubiquitination. Silencing FBXO45 alongside TRIM14 disruption attenuated the increased ZEB2 ubiquitination caused by TRIM14 inhibition. Moreover, overexpression of TRIM14 reduced ZEB2 ubiquitination, and forced expression of FBXO45 increased ZEB2 ubiquitination (Fig. 6f). Importantly, overexpression of TRIM14 together with FBXO45 abolished the increased ZEB2 ubiquitination caused by FBXO45 overexpression. Overall, these data further confirmed that TRIM14 increases the stability of ZEB2 by opposing FBXO45-mediated ubiquitination.

### TRIM14 function is proved in orthotopic nude mice model and GBM specimens

TRIM14 knockdown decreases the stability of ZEB2 and blocks glioblastoma cell invasion by mediating the proteasomal degradation of ZEB2, which was verified in LN229 and T98G cell lines. Further test should be induced in vivo. The LN229 cell transfected with shCtrl or shTRIM14 were transplanted in six pairs of orthotopic nude mice model (Fig. 7a). These findings were further confirmed by the survival curves, in which shTRIM14-transplanted xenografts exhibited significantly increased survival as compared with shCtrl-transplanted xenografts (***p < 0.001, *n* = 6, Fig. 7b). Bioluminescence images revealed that significant differences in the tumour volume between LN229 cells transduced with shCtrl and those cells transduced with shTRIM14, mice bearing LN229 cells transduced with shTRIM14 displayed a significant reduction compared with xenografts transduced with shCtrl (***p < 0.001, *n* = 3, Fig. 7c). HE-stained orthotopic xenograft tumors are given in Fig. 7d, cell motion was weaken in shTRIM14-transplanted groups. To explore the expression of TRIM14 and ZEB2 in the in orthotopic nude mice mode, we randomly selected four pairs mice from shCtrl-transplanted group and shCtrl-transplanted group. Western blot analysis demonstrated that TRIM14 and ZEB2 were highly expressed in shCtrl-transplanted group but showed significantly decreased expression in matched shCtrl-transplanted group (Fig. 7e). To validate the association between TRIM14 and ZEB2 in GBM patients, we performed IHC staining of these four proteins, a highly significant correlation between TRIM14 and ZEB2 was observed in these GBM specimens. Tumors with high level of TRIM14 tended to express high levels of ZEB2, whereas tumors with low level of TRIM14 tended to express low levels of ZEB2 (Fig. 7f).

**Fig. 7:** TRIM14 function was demonstrated in vivo and IHC. **a** ShCtrl-transplanted and shTRIM14-transplanted LN229 cells were counted and transplanted in orthotopic nude mice model respectively, *n* = 6. **b** Survival curve of shCtrl-transplanted or shTRIM14-transplanted intracranial xenografts. ***, *P* < 0.001, *n* = 6. **c** Representative pseudocolour bioluminescence images of orthotopic tumours bearing control or TRIM14-depleted LN229 cells on the days as indicated. Quantification of tumor volume is shown. ***p < 0.001; *n* = 3 experiment. **d** The HE assay was performed to show tumor cytostructure. **e** Western blot analysis of TRIM14 and ZEB2 extracted from four pairs mice from shCtrl-transplanted group and shCtrl-transplanted group. Equal loading is confirmed by β-actin levels. **f** IHC staining of TRIM14 and ZEB2 in four representative GBM specimens

## Discussion

The primary cause of mortality in patients with glioblastoma is metastasis, but the underlying mechanisms of tissue invasion and metastasis remain incompletely understood [36]. The TRIM family, which contains more than 70 members, has been identified as being involved in the progression, transformation, autophagy, and metastasis of cancer [37–39]. TRIM14 belongs to the TRIM protein family, and has been shown to be markedly increased in human osteosarcoma tissues and cell lines and strongly associated with aggressive characteristics and poor patient outcome [10, 14, 16, 40, 41]. However, the role played by TRIM14 in glioblastoma has not been completely confirmed.

Here we report the first demonstration that TRIM14 functions as a tumor invasion promoter in glioblastoma. Our findings demonstrate an increased expression levels of TRIM14 in glioblastoma, suggesting it functions as an oncogene and is involved in glioblastoma invasion. When we examined clinical glioblastoma tissues, we found that TRIM14 was upregulated in glioblastoma specimens at both the mRNA transcript and protein level. Consistent with this finding, TRIM14 expression levels were noticeably high in high-grade glioblastoma and several glioblastoma cell lines. Furthermore, functional tests showed that TRIM14 deletion significantly reduced cell invasion and migration ability. Additionally, we found this function was closely related to EMT. Deleting TRIM14 altered EMT biomarker levels: it downregulated N-cadherin and vimentin, and upregulated E-cadherin. Although the role of TRIM14 in vivo remains to be more tested in future studies, the marked impairment of wound healing and antagonism of the invasive growth of multiple glioblastoma cell lines induced by TRIM14 knockdown strongly support our hypothesis that TRIM14 promotes glioblastoma cell growth and invasion.

Zinc finger E-box binding homeobox 2 (ZEB2) is a transcription factor that regulates EMT [34, 42]. ZEB2 regulates cell proliferation, migration, invasion, and apoptosis in several forms of human cancer [43–47]. Importantly, ZEB2 is associated with tumorigenicity in glioblastoma [48]. Our data indicate that loss of TRIM14 downregulates ZEB2 by post-translational modification but not by transcriptional regulation. Moreover, we demonstrated for the first time that loss of TRIM14 promotes ZEB2 polyubiquitination and subsequent proteasomal degradation. TRIM14-induced EMT is dependent on ZEB2 to regulate EMT-associated biomarkers. These molecular events are consistent with our observation that TRIM14 is critical in modulating invasion and migration in glioblastoma through ZEB2. However, the specific mechanism by which ZEB2 polyubiquitination is altered by TRIM14 remains to be investigated.

In conclusion, TRIM14 expression may have significant value as an indicator of unfavorable progression for glioblastoma patients. We provide compelling evidence that decreased expression of TRIM14 inhibits cell migration and invasion through effects on EMT mediated via changes in ZEB2 stability.

## Conclusions

To the best of our knowledge, this is the first study to investigate the relationship between TRIM14 and ZEB2 in GBM, and our results shed light on that TRIM14 facilitates invasion and migration of GBM by means of delaying ZEB2 degradation. Thus, the TRIM14/ZEB2 axis was revealed an oncogenic function in GBM and this might be provided as a novel therapeutic target.

## Additional files

Additional file 1: **Figure S1.** TRIM14 is overexpression in GBM and correlates with poor prognosis. (A) The expression of TRIM14 was analyzed in control brain tissues and GBM tissues of the REMBRANDT (*P* < 0.0001, *n* = 227), GSE16011 (*P* = 0.0106, *n* = 284) and TCGA(P < 0.0001, *n* = 594) glioblastoma datasets. (B) Kaplan–Meier curves showing the overall survival of patients with high or low expression of TRIM14 in GBM patients using the REMBRANDT(*P* = 0.0469, *n* = 227), GSE16011 (*P* = 0.0340, *n* = 284) and TCGA databases(*P* = 0.0489, *n* = 594). (TIF 528 kb)

Additional file 2: **Figure S2.** TRIM14 promotes proliferation in glioma. (A) CCK-8 assay displays decreased proliferation in LN229 and U251 after silencing TRIM14. ***p < 0.001; *n* = 3 experiment. (B) LN229 and U251 were treated with the indicated shRNA and performed colony formation assay. Quantification of colony formation assay is shown. ***p < 0.001; *n* = 3 experiment. (C) CCK-8 assay displays decreased proliferation in HS683 and U87 after overexpressing TRIM14. ***p < 0.001; *n* = 3 experiment. (D) HS683 and U87 were treated with vector or TRIM14 and performed colony formation assay. Quantification of colony formation assay is shown. ***p < 0.001; *n* = 3 experiment. (TIF 2304 kb)

## Abbreviations

ATCC: American Type Culture Collection
EMT: Epithelial–mesenchymal transition
EMT-TFs: EMT-inducing transcription factors
FBXO45: F-Box protein 45
GBM: Glioblastoma multiforme
qRT-PCR: Quantitative reverse transcription-polymerase chain reaction
TRIM14: Tripartite motif-containing 14
ZEB2: Zinc finger E-box binding homeobox 2

## References

[1] Ballester LY, Wang Z, Shandilya S, Miettinen M, Burger PC, Eberhart CG, Rodriguez FJ, Raabe E, Nazarian J, Warren K, Quezado MM (2013). Morphologic characteristics and immunohistochemical profile of diffuse intrinsic pontine gliomas. Am J Surg Pathol.

[2] Giunti L, Pantaleo M, Sardi I, Provenzano A, Magi A, Cardellicchio S, Castiglione F, Tattini L, Novara F, Buccoliero AM, de Martino M, Genitori L, Zuffardi O, Giglio S (2014). Genome-wide copy number analysis in pediatric glioblastoma multiforme. Am J Cancer Res.

[3] Lim SK, Llaguno SR, McKay RM, Parada LF (2011). Glioblastoma multiforme: a perspective on recent findings in human cancer and mouse models. BMB Rep.

[4] Dejaegher J, De Vleeschouwer S, De Vleeschouwer S (2017). Recurring glioblastoma: A case for reoperation?. Glioblastoma.

[5] Nestler U, Lutz K, Pichlmeier U, Stummer W, Franz K, Reulen HJ, Bink A (2015). Anatomic features of glioblastoma and their potential impact on survival. Acta Neurochir.

[6] Guan X, Li J, Lu X, Dong Y, Chen W, Li X (2014). Expression, purification, crystallization and preliminary x-ray diffraction analysis of the c-terminal nhl domain of human trim2. Acta Crystallogr F Struct Biol Commun.

[7] Kanno Y, Watanabe M, Kimura T, Nonomura K, Tanaka S, Hatakeyama S (2014). Trim29 as a novel prostate basal cell marker for diagnosis of prostate cancer. Acta Histochem.

[8] Hatakeyama S (2017). Trim family proteins: roles in autophagy, immunity, and carcinogenesis. Trends Biochem Sci.

[9] Nenasheva VV, Kovaleva GV, Uryvaev LV, Ionova KS, Dedova AV, Vorkunova GK, Chernyshenko SV, Khaidarova NV, Tarantul VZ (2015). Enhanced expression of trim14 gene suppressed sindbis virus reproduction and modulated the transcription of a large number of genes of innate immunity. Immunol Res.

[10] Nie C, Zhang Z, Zheng J, Sun H, Ning Z, Xu G, Yang N, Qu L (2016). Genome-wide association study revealed genomic regions related to white/red earlobe color trait in the Rhode Island red chickens. BMC Genet.

[11] Wang T, Ren Y, Liu R, Ma J, Shi Y, Zhang L, Bu R (2017). Mir-195-5p suppresses the proliferation, migration, and invasion of oral squamous cell carcinoma by targeting trim14. Biomed Res Int.

[12] Wang X, Guo H, Yao B, Helms J (2017). Mir-15b inhibits cancer-initiating cell phenotypes and chemoresistance of cisplatin by targeting trim14 in oral tongue squamous cell cancer. Oncol Rep.

[13] Hai J, Zhu CQ, Wang T, Organ SL, Shepherd FA, Tsao MS (2017). Trim14 is a putative tumor suppressor and regulator of innate immune response in non-small cell lung cancer. Sci Rep.

[14] Wang F, Ruan L, Yang J, Zhao Q, Wei W (2018). Trim14 promotes the migration and invasion of gastric cancer by regulating epithelialtomesenchymal transition via activation of akt signaling regulated by mir1955p. Oncol Rep.

[15] Hu G, Pen W, Wang M. Trim14 promotes breast cancer cell proliferation by inhibiting apoptosis. Oncol Res. 2018. 10.3727/096504018X15214994641786.10.3727/096504018X15214994641786PMC784841729562956

[16] Xu G, Guo Y, Xu D, Wang Y, Shen Y, Wang F, Lv Y, Song F, Jiang D, Zhang Y, Lou Y, Meng Y, Yang Y, Kang Y (2017). Trim14 regulates cell proliferation and invasion in osteosarcoma via promotion of the akt signaling pathway. Sci Rep.

[17] Wang T, Xu L, Jia R, Wei J (2017). Mir-218 suppresses the metastasis and emt of hcc cells via targeting serbp1. Acta Biochim Biophys Sin Shanghai.

[18] Pramanik A, Vangara A, Viraka Nellore BP, Sinha SS, Chavva SR, Jones S, Ray PC (2016). Development of multifunctional fluorescent-magnetic nanoprobes for selective capturing and multicolor imaging of heterogeneous circulating tumor cells. ACS Appl Mater Interfaces.

[19] Yilmaz M, Christofori G (2009). Emt, the cytoskeleton, and cancer cell invasion. Cancer Metastasis Rev.

[20] Sannino G, Marchetto A, Kirchner T, Grunewald TGP (2017). Epithelial-to-mesenchymal and mesenchymal-to-epithelial transition in mesenchymal tumors: a paradox in sarcomas?. Cancer Res.

[21] Drachsler M, Kleber S, Mateos A, Volk K, Mohr N, Chen S, Cirovic B, Tuttenberg J, Gieffers C, Sykora J, Wirtz CR, Mueller W, Synowitz M, Martin-Villalba A (2016). Cd95 maintains stem cell-like and non-classical emt programs in primary human glioblastoma cells. Cell Death Dis.

[22] Chaffer CL, San Juan BP, Lim E, Weinberg RA (2016). Emt, cell plasticity and metastasis. Cancer Metastasis Rev.

[23] Shibue T, Weinberg RA (2017). Emt, cscs, and drug resistance: the mechanistic link and clinical implications. Nat Rev Clin Oncol.

[24] Imani S, Hosseinifard H, Cheng J, Wei C, Fu J (2016). Prognostic value of emt-inducing transcription factors (emt-tfs) in metastatic breast cancer: a systematic review and meta-analysis. Sci Rep.

[25] Wels C, Joshi S, Koefinger P, Bergler H, Schaider H (2011). Transcriptional activation of zeb1 by slug leads to cooperative regulation of the epithelial-mesenchymal transition-like phenotype in melanoma. J Invest Dermatol.

[26] Casas E, Kim J, Bendesky A, Ohno-Machado L, Wolfe CJ, Yang J (2011). Snail2 is an essential mediator of twist1-induced epithelial mesenchymal transition and metastasis. Cancer Res.

[27] Drago-Garcia D, Espinal-Enriquez J, Hernandez-Lemus E (2017). Network analysis of emt and met micro-rna regulation in breast cancer. Sci Rep.

[28] Tang Y, Weiss SJ (2017). Snail/slug-yap/taz complexes cooperatively regulate mesenchymal stem cell function and bone formation. Cell Cycle.

[29] Caramel J, Papadogeorgakis E, Hill L, Browne GJ, Richard G, Wierinckx A, Saldanha G, Osborne J, Hutchinson P, Tse G, Lachuer J, Puisieux A, Pringle JH, Ansieau S, Tulchinsky E (2013). A switch in the expression of embryonic emt-inducers drives the development of malignant melanoma. Cancer Cell.

[30] Goossens S, Vandamme N, Van Vlierberghe P, Berx G (2017). Emt transcription factors in cancer development re-evaluated: beyond emt and met. Biochim Biophys Acta Rev Cancer.

[31] De Craene B, Berx G (2013). Regulatory networks defining emt during cancer initiation and progression. Nat Rev Cancer.

[32] Hegarty SV, Sullivan AM, O'Keeffe GW (2015). Zeb2: a multifunctional regulator of nervous system development. Prog Neurobiol.

[33] Bui TT, Nitta RT, Kahn SA, Razavi SM, Agarwal M, Aujla P, Gholamin S, Recht L, Li G (2015). Gamma-glutamyl transferase 7 is a novel regulator of glioblastoma growth. BMC Cancer.

[34] Li H, Mar BG, Zhang H, Puram RV, Vazquez F, Weir BA, Hahn WC, Ebert B, Pellman D (2017). The emt regulator zeb2 is a novel dependency of human and murine acute myeloid leukemia. Blood.

[35] Xu Y, Lee DK, Feng Z, Xu Y, Bu W, Li Y, Liao L, Xu J (2017). Breast tumor cell-specific knockout of twist1 inhibits cancer cell plasticity, dissemination, and lung metastasis in mice. Proc Natl Acad Sci U S A.

[36] Aroui S, Aouey B, Chtourou Y, Meunier AC, Fetoui H, Kenani A (2016). Naringin suppresses cell metastasis and the expression of matrix metalloproteinases (mmp-2 and mmp-9) via the inhibition of erk-p38-jnk signaling pathway in human glioblastoma. Chem Biol Interact.

[37] Esposito D, Koliopoulos MG, Rittinger K (2017). Structural determinants of trim protein function. Biochem Soc Trans.

[38] Jiang MX, Hong X, Liao BB, Shi SZ, Lai XF, Zheng HY, Xie L, Wang Y, Wang XL, Xin HB, Fu M, Deng KY (2017). Expression profiling of trim protein family in thp1-derived macrophages following tlr stimulation. Sci Rep.

[39] Ozato K, Shin DM, Chang TH, Morse HC (2008). Trim family proteins and their emerging roles in innate immunity. Nat Rev Immunol.

[40] Yu GH, Li AM, Li X, Yang Z, Peng H (2017). Bispecific antibody suppresses osteosarcoma aggressiveness through regulation of nf-kappab signaling pathway. Tumour Biol.

[41] Chen M, Meng Q, Qin Y, Liang P, Tan P, He L, Zhou Y, Chen Y, Huang J, Wang RF, Cui J (2016). Trim14 inhibits cgas degradation mediated by selective autophagy receptor p62 to promote innate immune responses. Mol Cell.

[42] Wang T, Chen X, Qiao W, Kong L, Sun D, Li Z (2017). Transcription factor e2f1 promotes emt by regulating zeb2 in small cell lung cancer. BMC Cancer.

[43] Eggers JC, Martino V, Reinbold R, Schafer SD, Kiesel L, Starzinski-Powitz A, Schuring AN, Kemper B, Greve B, Gotte M (2016). Microrna mir-200b affects proliferation, invasiveness and stemness of endometriotic cells by targeting zeb1, zeb2 and klf4. Reprod BioMed Online.

[44] Yue S, Wang L, Zhang H, Min Y, Lou Y, Sun H, Jiang Y, Zhang W, Liang A, Guo Y, Chen P, Lv G, Wang L, Zong Q, Li Y (2015). Mir-139-5p suppresses cancer cell migration and invasion through targeting zeb1 and zeb2 in gbm. Tumour Biol.

[45] Depner C, Zum Buttel H, Bogurcu N, Cuesta AM, Aburto MR, Seidel S, Finkelmeier F, Foss F, Hofmann J, Kaulich K, Barbus S, Segarra M, Reifenberger G, Garvalov BK, Acker T, Acker-Palmer A (2016). Ephrinb2 repression through zeb2 mediates tumour invasion and anti-angiogenic resistance. Nat Commun.

[46] Jiang M, Zhong T, Zhang W, Xiao Z, Hu G, Zhou H, Kuang H (2017). Reduced expression of mir2055p promotes apoptosis and inhibits proliferation and invasion in lung cancer a549 cells by upregulation of zeb2 and downregulation of erbb3. Mol Med Rep.

[47] Wu X, Yan T, Wang Z, Wu X, Cao G, Zhang C (2017). Lncrna zeb2-as1 promotes bladder cancer cell proliferation and inhibits apoptosis by regulating mir-27b. Biomed Pharmacother.

[48] Sailer MH, Sarvepalli D, Bregere C, Fisch U, Guentchev M, Weller M, Guzman R, Bettler B, Ghosh A, Hutter G. An enzyme- and serum-free neural stem cell culture model for emt investigation suited for drug discovery. J Vis Exp. 2016;(114). 10.3791/54018.10.3791/54018PMC509194827583933

